This article has been retracted.

# Expression of CDK6 in Stomach Cancer and the Effect of CDK4/6 Inhibitor PD-0332991 on the Function of Stomach Cancer Cells

**DOI:** 10.1155/2022/2402567

**Published:** 2022-04-30

**Authors:** Yu Liu, Yan Zhao, Chongxu Han, Chuanli Ren

**Affiliations:** ^1^Department of Laboratory Medicine, School of Medicine of Yangzhou Univerisity, Yangzhou, Jiangsu Province, China 225000; ^2^Medical Research Center, Clinical Medical College, Yangzhou University, Yangzhou, Jiangsu Province, China 225000; ^3^Department of Laboratory Medicine, Clinical Medical College, Yangzhou University, Yangzhou, Jiangsu Province, China 225000

## Abstract

**Objective:**

To study the expression and prognostic value of CDK6 in stomach cancer and the function of CDK4/6 inhibitor PD-0332991 on the proliferation of stomach cancer cells.

**Methods:**

Immunohistochemistry was used to detect the expression of CDK6 in stomach cancer tissues and adjacent normal tissues and to analyze the effect of CDK6 on clinicopathological parameters of stomach cancer patients. Kaplan-Meier plotter was employed to study the relationship between CDK6 and overall survival in stomach cancer. Western blot and RT-PCR were used to detect protein and gene expression of CDK6 in different cells. The effects of CDK4/6 inhibitor PD-0332991 on apoptosis and aging of stomach cancer cells were detected by flow cytometry and *β*-galactosidase aging staining assay. The effects of CDK4/6 inhibitor PD-0332991 on the invasion and migration of stomach cancer cells were explored by the wound healing experiment and the Transwell experiment. The supernatant of stomach cancer cells was collected, and the effect of CDK4/6 inhibitor PD-0332991 on tumor markers of stomach cancer cells was detected by biochemical immunoassay.

**Results:**

(1) CDK6 was highly expressed in stomach cancer tissues and cells. (2) Abnormally elevated CDK6 expression results in shorter survival in stomach cancer patients. (3) CDK4/6 inhibitor PD-0332991 could block the proliferation of stomach cancer cells, but not stomach epithelial proliferation. PD-0332991 could inhibit the secretion of pro-GRP by MGC 823. (4) PD-0332991 could advance the development of the apoptosis and senescence of stomach cancer cells and suppressed the invasion and migration of stomach cancer cells.

**Conclusion:**

CDK6 expression is elevated in gastric cancer, and the CDK4/6 inhibitor PD-0332991 can remarkably promote apoptosis and senescence of stomach cancer cells and effectively inhibit the migration and invasion of stomach cancer cells.

## 1. Introduction

Globally, stomach cancer is the fourth most common malignancy and the second leading cause of mortality [1]. Environmental factors, Helicobacter pylori infection, smoking, and lifestyle play major roles in stomach cancer. At present, although the research on gastric cancer has achieved great success, the molecular mechanism of gastric cancer is still not fully understood, and the effective treatment of gastric cancer is still a hot issue [2, 3]. Abnormal expression of CDK6 affects the initiation and progression of various malignant tumors [4]. One of the hallmarks of cancer is cell cycle disorder that leads to abnormal cell proliferation. Drugs targeting the cell cycle are ideal for tumor-targeted therapy [5]. Targeting CDK4/6 therapy is currently a hot spot in the development of antitumor drugs. It mainly acts by inhibiting cell cycle kinases, inhibiting the process of the G1 phase to S phase, and then inhibiting the proliferation of tumor cells. FDA approves palbociclib, ribociclib, and abemaciclib for breast cancer [6, 7]. Compared to other cell cycle inhibitors, these drugs are generally well tolerated. Extensive preclinical evidence shows that CDK4/6 inhibitors are widely used in several types of tumors including triple-negative breast cancer, non-small-cell lung cancer, melanoma, and head and neck squamous cell carcinoma [8]. Currently, there are at least 100 clinical trials underway in various tumor types, but the role of targeting CDK4/6 in stomach cancer is still unclear [9]. In this research, we explored the expression level of CDK6 in stomach cancer and the regulation of CDK4/6 inhibitor PD-0332991 on stomach cancer cell proliferation, aimed at providing more promising targets for stomach cancer.

## 2. Method

### 2.1. Research Objects and Clinical Data

Stomach cancer tissue chips (HStm-Ade180Sur-04) were obtained from Shanghai Xinchao Biotechnology Co., Ltd. (Shanghai, China) and included stomach cancer tissues and matched adjacent normal tissues from 90 patients.

### 2.2. Cell Line Culture

Human stomach cancer cells BGC-823, AGS, SNU1, MKN45, MKN1, MGC-803, HGC-27, SGC-7901, and stomach normal cell GES-1 were obtained from Shanghai Institutes for Biological Sciences, Chinese Academy of Sciences. BGC-823, SNU1, MKN45, MKN1, MGC-803, HGC-27, SGC-7901, and GES-1 were routinely cultured in the RPMI 1640 medium. AGS was cultured in Ham's F-12 medium. Both RPMI1640 medium and Ham's F-12 medium contain 10% FBS and 1% penicillin and streptomycin. All cells were cultured in an incubator at 37°C and 5% CO_2_.

### 2.3. Immunohistochemical Staining

A significantly representative tumor region was selected from the HE-stained sections with caution. Deparaffinization in xylene and graded ethanol, heat retrieval of antigen, 0.3% hydrogen peroxide to restrain endogenous peroxidase, and serum incubation to inhibit nonspecific binding. Sections were incubated with CDK6 antibody for 24 h. Specimens were incubated with secondary antibodies labeled with biotin and avidin labeled with horseradish peroxidase and stained by the DAB method. Patient sections were independently assessed by 2 physicians. The staining intensity is randomly divided into 4 grades: 0-3 grades correspond to no, weak, moderate, or strong staining, respectively. The formula for determining positive staining was as follows: total score = positive percentage score × strength. A score of <2 points was scored as “negative”, and a score of ≥2 was scored as “positive.”

### 2.4. RT-qPCR Detection

Total RNA was extracted from cells and reverse transcribed into cDNA. PCR was performed using SYBR Green reagents and primers. CDK6 primer sequences are as follows: upstream: 5′-CAAGATCTCTGAGGAGTACGTGGGCCTGT-3′. downstream 5′-GCGGTACCTGTCTCAGAAGGTGCATTCT-3′.

Suitable reaction conditions were chosen. GAPDH was used as an internal reference.

### 2.5. Western Blot Detection

Total protein extracted from cells was quantified. Electrophoresis was performed first and then transferred to a polyvinylidene fluoride (PVDF) membrane. PVDF membranes were blocked with 5% nonfat milk and incubated with primary antibodies overnight. Primary antibodies were rabbit anti-CDK6 (1 : 1000) and rabbit anti-GAPDH (1 : 5000). The membrane was washed 3 times with TBS-Tween solution and then incubated with secondary antibody. The membrane was washed three times with TBS-Tween solution and finally developed by the ECL method.

### 2.6. CCK-8 Detection and *β*-Galactosidase Cell Senescence Staining

The cells were adjusted to an appropriate concentration and seeded in a 96-well plate at 3000 cells per well. After adding the appropriate concentration of PD-0332991 and incubating for 48 h and 72 h, the absorbance value was measured and recorded on the cell growth curve, and IC50 was calculated. For *β*-galactosidase senescence stain, drug-treated cells were collected and fixed with fixative. Stain according to the staining kit instructions and then take pictures using an inverted microscope. The experiment was repeated three times.

### 2.7. Detection of Apoptosis by AnnexinV-FITC/PI Double Staining

The collected drug-treated stomach cells were suspended in 500 *μ*l of buffer, labeled with 5 *μ*l of FITC-Annexin V reagent and 5 *μ*l of propidium iodide, and then rapidly detected by flow cytometry within 1 h. The apoptotic rate was expressed as the percentage of apoptotic cells in Annexin V+/PI- and Annexin V+/PI+ quadrants, and each sample were repeated three times.

### 2.8. Cell Migration Ability and Invasion

For cell invasion, assays were performed using Matrigel-coated Transwell chambers. Drug-treated cells were resuspended in a 200 *μ*l medium without FBS and seeded in the upper chamber. The lower chamber is a medium containing 10% FBS.

For cell migration, a chamber without Matrigel matrix was used and other steps were the same as for the invasion assay. The migration ability and the invasion ability were all carried out under the condition of 37°C, and 5 predetermined fields of view (×200) were photographed under the microscope. For wound healing experiment, we inoculate cells with a six-well plate, add drugs for 72 hours, draw even traces with a 100 *μ*l pipette tip perpendicular to the bottom of the six-well plate, take pictures under an inverted microscope, and add 2% bovine serum-containing medium to continue. Photographs were taken again after 24 h of culture. Each sample was replicated three times.

For wound healing experiment, the cells were seeded into a six-well plate and incubated with drugs for 72 hours. Perpendicular to the bottom of the plate, we use 100*μ*l to draw uniform marks on the tip of the pipette, take photos under an inverted microscope, and add 2% medium containing bovine serum. After incubation for 24 hours, we take photos again. Each sample was repeated more than 3 times.

### 2.9. Determination of Cell-Secreted Tumor Markers

The supernatants of stomach cancer cells in the drug-treated and control group were collected, respectively, and tumor markers were tested by biochemical immunoassay as soon as possible.

### 2.10. Statistical Analysis

All data were statistically analyzed using SPSS 20.0. The enumeration data were expressed by the number of cases, and the chi-square (*χ*^2^) test was used. *p* < 0.05 was considered statistically meaningful.

## 3. Results

### 3.1. Expression of CDK6 in Stomach Cancer

Immunohistochemical staining brought to light that the expression level of CDK6 was notably elevated in stomach cancer tissues compared with normal tissues (*p* = 0.0066) (Figures 1(a) and 1(b)). CDK6 mainly exists in the cytoplasm of stomach cancer cells. The expression levels of CDK6 mRNA in MKN1, AGS, SNU-1, and MKN45 were 2.36 ± 0.13, 3.69 ± 0.20, 5.39 ± 0.23, and 4.13 ± 0.21, respectively. Compared with GSE-1 cells, the expression of CDK6 mRNA in stomach cancer cells was increased, as shown in Figure 1(c). The results of Western blot detection were similar to the RT-qPCR trend (Figures 1(d) and 1(e)). We used the Kaplan-Meier plotter to study the relationship between CDK6 and overall survival in stomach cancer patients. The Kaplan-Meier plotter contains survival information of 875 stomach cancer patients from TCGA, EGA, and GEO databases. It can be used to study the effect of single factors on survival time. The data were calculated according to hazard ratios (HRs) and log-rank *p* values. The CDK6-positive patients had a lower survival rate compared to the CDK6-negative group, *p* < 0.0001 (Figure 1(f)).

### 3.2. Influence of CDK6 Expression on Clinicopathological Parameters of Patients

Univariate analysis revealed that the positive expression of CDK6 has relation with the age in stomach cancer (*p* = 0.014), but not with sex, tumor diameter, tumor stage, AJCC stage, and lymph node metastasis (*p* > 0.05), as shown in Table 1.

### 3.3. Effects of PD-0332991 on Proliferation and Secretion of Tumor Markers in Stomach Cancer Cells

We used CCK8 to detect whether the stomach cancer cell line PD-0332991 had an inhibitory effect on SNU1, AGS, NKN1, and MKN45. The results showed that the IC_50_ of PD-0332991 for SNU1, AGS, NKN1, and MKN45 at 48 hours and 72 hours were 80.17 nM and 61.12 nM, 6265 nM and 4984 nM, 31780 nM and 2417 nM, and 31780 nM and 24170 nM, respectively; but for GES-1, its IC_50_ was undetectable. This indicated that PD-0332991 could block the growth of stomach cancer cells in a time- and concentration-dependent manner. Figures 2(a)-–2(d) are growth curves of the inhibition effect of different concentrations of PD-0332991 on stomach cancer cells. BGC-823 cells were incubated with PD-0332991 (0, 5, and 10 *μ*M) for 48 h, and the supernatants before and after drug treatment were collected to detect the changes of CA12-5, CEA, CA19-9, HE4, CA72-4, and pro-GRP. The results showed that different concentrations of PD-0332991 could inhibit the secretion of pro-GRP by BGC-823 in a concentration-dependent manner, as shown in Figure 2(e). But different concentrations of PD-0332991 seemed to not affect the expression of BGC-823 CA72-4. After PD-0332991 treated BGC-823, the secretion of CA12-5, CEA, CA19-9, and HE4 were all lower than the lower limit of the detection range of the detector, and the specific values could not be measured.

### 3.4. Effects of PD-0332991 on Apoptosis, Senescence, Invasion, and Migration of Stomach Cancer Cells

To deeply study the effect of PD-0332991 on the senescence of stomach cancer cells, AGS and MKN45 were selected as experimental objects in this experiment, and PD-0332991 was used at an appropriate concentration for 72 hours, and then, the cells were collected for *β*-galactosidase staining to detect their senescence. Our experimental results revealed that PD-0332991 could induce senescence in AGS and MKN45 (Figures 3(a) and 3(b)).

To test whether PD-0332991 can induce apoptosis of stomach cancer cells, 5 *μ*M PD-0332991 was selected in this experiment to act on MGC-803, HGC-27, BGC-823, SGC-7901, and AGS for 48 h, respectively. The experimental cells were labeled with FITC-labeled Annexin V and PI, and the apoptosis of stomach cancer cells was tested by flow cytometry. The experimental results showed that 5 *μ*M PD-0332991 could induce the apoptosis of MGC-803, HGC-27, and SGC-7901, but 5 *μ*M PD-0332991 did not seem to promote the apoptosis of BGC-823 cells, as shown in Figure 3(c).

Based on the above experimental results, PD-0332991 can induce apoptosis and senescence of stomach cancer cells. To deeply study the effect of PD-0332991 on migration and invasion of stomach cancer cells, AGS and SNU1 were selected as experimental objects in this experiment. AGS and SNU1 were incubated with PD-0332991 at 5000 nM and 100 nM for 72 hours, respectively, and then, the cells were collected for Transwell and wound healing experiments to detect the effects of drugs on invasion and migration. In summary, PD-0332991 could notably inhibit the migration and invasion ability of AGS and SNU1 after 72h treatment, as shown in Figures 3(d)–3(g).

## 4. Discussion

Stomach cancer is one of the malignant tumors that threaten the life and health of Chinese residents. However, the incidence and mortality of stomach cancer are still increasing [10]. Surgical resection of tumor tissue is still an effective method for stomach cancer. However, due to the lack of effective early diagnosis methods, the best operation time is often missed when stomach cancer is diagnosed, resulting in a very low 5-year survival rate. Due to the heterogeneity of gastric cancer, there are no particularly effective targeted drugs at present. Patients can only rely on adjuvant therapy such as radiotherapy and chemotherapy to prolong their life, but the effect is relatively poor [10–12]. Therefore, the development of new targeted therapy drugs for stomach cancer has important clinical significance.

CDK6 acts as an oncogene in a variety of cancers, but there are few studies in stomach cancer. This study found that compared with adjacent normal tissues, CDK6 was elevated in stomach cancer tissues, and the expression of CDK6 protein and gene in stomach cancer cells was also remarkably higher than that in GES-1. The increased expression level of CDK6 was positively related to the poor prognosis of patients with stomach cancer. Then, we treated stomach cancer cells with the PD-0332991. The results of CCK-8 detection revealed the stomach cancer cells MKN45, MKN1, AGS, and SNU1 were more sensitive to PD-0332991, but PD-0332991 had no effect on the growth of GES-1. PD-0332991 can inhibit the secretion of pro-GRP by BGC-823. Flow cytometric apoptosis detection and *β*-galactosidase senescence staining showed that PD-0332991 could effectively promote apoptosis and senescence, thereby inhibiting the proliferation of stomach cancer cells. We also found that PD-0332991 could significantly block the invasion and migration of stomach cancer cells.

CDK4 and CDK6 are core drivers of the cell cycle and are critical in the initiation and development of various malignancies tumors. Angiogenesis has an important effect on tumorigenesis and is controlled by platelet-derived growth factor (PDGF) and vascular endothelial growth factor (VEGF) [13, 14]. Studies have reported that the PI3K/Akt signaling is cocontrolled by VEGF and PDGF [15]. Depending on PI3K/Akt signal, VEGF induces the proliferation of neuroblastoma and PDGF affects the migration of colon cancer cells [16]. Abnormally activated PI3K/Akt signaling pathway can block apoptosis, promote cell cycle progression, and accelerate cell proliferation. This pathway is also involved in angiogenesis and tumor formation and acts as an important part of tumor invasion and metastasis. Therefore, we speculate that CDK4/6 inhibitors can suppress the growth and metastasis of stomach cancer by blocking VEGF and its downstream signaling. However, there are still have some shortcomings in this study. This study only studied the expression and prognostic value of CDK6 in gastric cancer and the effect of the CDK4/6 inhibitor PD-0332991 on the proliferation of gastric cancer cells [17]. The specific mechanism of the effect of the CDK4/6 inhibitor PD-0332991 on the proliferation of gastric cancer cells has not been studied in-depth, so we will further study this in the future.

In summary, this research found that the expression of CDK6 is elevated in stomach cancer, and the abnormal increase of CDK6 can lead to a poor prognosis of stomach cancer patients. The CDK4/6 inhibitor PD-0332991 can promote stomach cancer cell apoptosis and senescence and inhibit stomach cancer cell migration and invasion.

## Figures and Tables

**Figure 1:** Expression of CDK6 in stomach cancer. (a, b) Expression of CDK6 in stomach cancer tissues. (c) Expression of CDK6 mRNA in stomach cancer cells and stomach epithelial cells. (d, e) Expression of CDK6 protein in stomach cancer cells and stomach epithelial cells. (f) The effect of CDK6 on the overall productivity of stomach cancer patients.

**Figure 2:** The effect of PD-0332991 on the proliferation of stomach cancer cells. (a–d) The growth curves of the inhibition effects of PD-0332001 on SNU-1, AGS, MKN45, and MKN1, respectively. (e) The effect of PD-0332991 on the secretion of pro-GRP by BGC-823.

**Figure 3:** Effects of PD-0332991 on senescence, apoptosis, migration, and invasion of stomach cancer cells. (a, b) PD-0332991 promotes stomach cancer cell senescence. (c) PD-0332991 promotes stomach cancer cell apoptosis. (d–g) PD-0332991 inhibits stomach cancer cell invasion and migration.

**Table 1:** Effects of CDK6 expression on clinicopathological characteristics of patients.

Metric	CDK6 positive (*n* = 31)	CDK6 negative (*n* = 59)	*χ* ^2^ value	*p* value
Sex			1.489	0.222
Man	24	45		
Woman	7	14		
Age			6.001	0.014
<60 years old	6	21		
The 60-year-old oneself	25	38		
Tumor diameter			1.795	0.18
<5 cm	15	20		
≥5 cm	16	39		
Tumor stage			2.45	0.118
I+II	11	12		
III+IV	20	47		
AJCC by stages			1.034	0.309
I-II	15	22		
III-IV	16	37		
T by stages			0.02	0.886
T1+T2	4	7		
T3+T4	27	52		
Lymphatic metastasis			0.029	0.865
N0	10	18		
N1-3	21	41		

## Data Availability

No data were used to support this study.
